# Photosynthetic Responses to Heat Treatments at Different Temperatures and following Recovery in Grapevine (*Vitis amurensis* L.) Leaves

**DOI:** 10.1371/journal.pone.0023033

**Published:** 2011-08-26

**Authors:** Hai-Bo Luo, Ling Ma, Hui-Feng Xi, Wei Duan, Shao-Hua Li, Wayne Loescher, Jun-Fang Wang, Li-Jun Wang

**Affiliations:** 1 Beijing Key Laboratory of Viticulture and Enology, and Key Laboratory of Plant Resource Science, Institute of Botany, Chinese Academy of Sciences, Beijing, People's Republic of China; 2 Graduate University of Chinese Academy of Sciences, Beijing, People's Republic of China; 3 Key Laboratory of Plant Germplasm Enhancement and Speciality Agriculture, Wuhan Botanical Garden, Chinese Academy of Sciences, Wuhan, People's Republic of China; 4 College of Agriculture and Natural Resources, Michigan State University, East Lansing, Michigan, United States of America; Cairo University, Egypt

## Abstract

**Background:**

The electron transport chain, Rubisco and stomatal conductance are important in photosynthesis. Little is known about their combined responses to heat treatment at different temperatures and following recovery in grapevines (*Vitis spp.*) which are often grown in climates with high temperatures.

**Methodology/Findings:**

The electron transport function of photosystem II, the activation state of Rubisco and the influence of stomatal behavior were investigated in grapevine leaves during heat treatments and following recovery. High temperature treatments included 35, 40 and 45°C, with 25°C as the control and recovery temperature. Heat treatment at 35°C did not significantly (*P*>0.05) inhibit net photosynthetic rate (*P*_n_). However, with treatments at 40 and 45°C, *P*_n_ was decreased, accompanied by an increase in substomatal CO_2_ concentration (*C*_i_), decreases in stomatal conductance (*g*_s_) and the activation state of Rubisco, and inhibition of the donor side and the reaction center of PSII. The acceptor side of PSII was inhibited at 45°C but not at 40°C. When grape leaves recovered following heat treatment, *P*_n_, g_s_ and the activation state of Rubisco also increased, and the donor side and the reaction center of PSII recovered. The increase in *P*_n_ during the recovery period following the second 45°C stress was slower than that following the 40°C stress, and these increases corresponded to the donor side of PSII and the activation state of Rubisco.

**Conclusions:**

Heat treatment at 35°C did not significantly (*P*>0.05) influence photosynthesis. The decrease of *P*_n_ in grape leaves exposed to more severe heat stress (40 or 45°C) was mainly attributed to three factors: the activation state of Rubisco, the donor side and the reaction center of PSII. However, the increase of *P*_n_ in grape leaves following heat stress was also associated with a stomatal response. The acceptor side of PSII in grape leaves was responsive but less sensitive to heat stress.

## Introduction

High temperature negatively affects plant growth and survival and hence crop yield. Photosynthesis is known to be one of the most heat-sensitive processes, and it can be inhibited by high temperature before other symptoms of stress are detected [1], [2]. Inhibition of photosynthesis by heat stress has long been attributed to an impairment of electron transport activity, especially the inhibition of photosystem II (PSII) activity [3], [4]. Heat stress not only damages the oxygen-evolving complex of PSII [5], [6], but also impairs electron transfer within the PSII reaction centres [7], [8], [9] and downstream of PSII. Some authors [10], [11] have suggested that the initial site of the inhibition is associated with a Calvin cycle reaction, especially inactivation of Rubisco [12], [13], [14], [15]. However, for different species, the specific effects of heat stress maybe different.

Worldwide, grape has become one of the most productive and important specialty crops. In many production regions, the maximum midday air temperature can reach more than 40°C, which is especially critical at berry ripening. Some researchers suggested the optimum temperature for photosynthesis is between 25°C and 35°C for some grape cultivars [16], [17]. Temperatures above 35°C generally reduce photosynthesis in grape leaves. Climate change may produce more frequent high temperature conditions close to the current northern limit of grape cultivation [18]. Extreme temperatures may therefore endanger berry quality and economic returns [19]. Although there are many reports dealing with the influence of heat stress to photosynthesis in grape leaves [20], [21], [22], [23], a very limited number of papers consider the combined response of the components of PSII, Rubisco and stomatal conductance to heat stress [24], [25]. Recently, Kadir [24] and Kadir et al. [25] determined the response of *Vitis* species to high temperature under controlled environmental conditions through chlorophyll fluorescence measurements such as F_v_/F_m_, F_v_ and F_o_. It is not known if inhibition of grape photosynthesis by heat stress is caused by an impairment of electron transport or Rubisco activity. Moreover, the effect of heat on the donor side, acceptor side, reaction center, and on energy partitioning of PSII in grapevine is not clear. In contrast, studies about effects of low temperatures on photosynthetic performance of grape leaves from electron transport and energy partitioning are relatively abundant [23], [26], [27]. In addition, recovery from heat stress is an important factor of heat tolerance in plants. Plants, including grapevine, may be most likely to experience heat stress around midday, and relatively normal temperatures otherwise. Thus, plants may be exposed to a heat stress – recovery – heat stress – recovery cycle. However, less information is available on the plant behavior under the heat-stress recovery compared with under heat stress. In the past, attention usually was focused on the plant's direct response to stress. Consequently, more definitive studies on the plant traits for heat tolerance must be conducted to understand the mechanism of the recovery from heat. These results may help develop modern and acceptable technologies to increase and stabilize berry yield and qualities.

Inhibition of PSII leads to a decrease in variable chlorophyll fluorescence. Thus, in vivo chlorophyll fluorescence may be used to detect changes in the photosynthetic apparatus [28], [29]. Strasser *et al.* have developed a method for the analysis of the kinetics of fast fluorescence increases since the non-destructive measurements can be done with a high resolution of 10 µs [30]. All oxygenic photosynthetic materials investigated so far show a polyphasic fluorescence rise consisting of a sequence of phases, denoted as O, J, I, and P (OJIP test). With this test, it is possible to calculate several phenomenological and biophysical expressions of PSII. The kinetics of OJIP are considered to be determined by changes in the redox state of Q_A_, but at the same time, the OJIP transient reflects the reduction of the photosynthetic electron transport chain [31]. The OJIP test has been a powerful tool for the *in vivo* investigation of the behavior of PSII function including energy absorption, trapping, and electron transport [30], [32], [33].

In the present study, gas exchange parameters, chlorophyll fluorescence parameters and the activity state of Rubisco in grape leaves during high temperature (35, 40 or 45°C) treatments and following recovery (stress-recovery-stress-recovery) were investigated. Our objective was to determine the importance of electron transport, Rubisco and stomatal factors to maintain photosynthesis and the sensitivity of components of the photosynthetic apparatus in grape leaves under high temperature stress and during recovery.

## Results

### Net photosynthesis rate (*P*_n_), substomatal CO_2_ concentration (*C*_i_) and stomatal conductance (*g*_s_)

At normal growth conditions of 25°C, *P*_n_, *C*_i_ and *g*_s_ of grape leaves did not change during the experiment (over the 3 days of the growth period monitored). Heat stresses at 35°C at two times did not significantly (*P*>0.05) influence *P*_n_, *C*_i_ and *g*_s_ of grape leaves compared with the control (at 25°C). A decline of *P*_n_ and *g*_s_ after 40 and 45°C treatments was observed, accompanied with a *C*_i_ increase. Heat stress at 45°C had stronger negative impact on *P*_n_ and *g*_s_ than 40°C and recovered more slowly. On the fourth day of recovery (Day 6) after the second heat stress, *P*_n_, *C*_i_ and *g*_s_ of plants that had received a 40°C treatment recovered to the control levels, but those exposed to 45°C were still exhibiting an effect of heat stress (Fig. 1).

**Figure 1:** *P*_n_, *C*_i_ and g_s_ in grape leaves under different heat treatments and following recovery. 25°C: normal growth and recovery temperature; 35, 40 and 45°C: high temperature treatments. Each value represents the mean ± S.E. of four replicates. At the same time point, the numerical values with different letters are significantly different (*P*<0.05) according to Duncan's multiple comparison.

### Donor side, reaction centre and acceptor side of PSII and PSI

It has been shown that heat stress can induce a rapid rise in the OJIP polyphasic fluorescence transients. This phase, occurring at around 300 µs and labeled K, is caused by an inhibition of the oxygen evolving complex (OEC). The amplitude of step K can therefore be used as a specific indicator of damage to PSII donor side [26]. Fig. 2 shows the changes in the amplitude in the K step expressed as the ratio W_K_. Compared with the control (25°C), heat stress at 35°C did not alter W_K_ of grape leaves. After the first heat treatment of 40°C or 45°C for 5 h, W_K_ of grape leaves increased steeply, and W_K_ was higher at 45°C than at 40°C. During the following recovery (on Day 2), W_K_ values of these treatments were similar to the control level. However, they rapidly increased again after the second heat stress. On the first day of recovery (Day 3), they declined to some extent, but W_K_ of the 45°C treatment was bigger than that of the 40°C treatment. On the fourth day of recovery (Day 6), W_K_ of the 40°C and 45°C treatments recovered to the control level.

**Figure 2:** Donor side (W_K_) and reaction center (RC_QA_) parameters of PSII in grape leaves under different heat treatments and following recovery. *W*_k_ = (*F*_k_−*F*_o_)/(*F*_j_−*F*_o_); RC_QA_ = *ϕ*_Po_×(V_j_/*M*_o_)×(ABS/CS). The definition of these parameters is shown in detail in Table 2. 25°C: normal growth and recovery temperature; 35, 40 and 45°C: high temperature treatments. Each value represents the mean ± S.E. of four replicates. At the same time point, the numerical values with different letters are significantly different (*P*<0.05) according to Duncan's multiple comparison.

RC_QA_ shows the density of the of Q_A_-reducing PSII reaction centers. Fig. 2 demonstrates that heat stress at 35°C did not influence the RC_QA_ during the experiment. The first (on Day 1) and second (on Day 2) stresses of 40°C or 45°C significantly (*P*<0.05) reduced the RC_QA_. The RC_QA_ values of the two treatments returned to control values during the first recovery. After the second stress, RC_QA_ values of the two treatments basically reached the level of controls during recovery of the first day.

Fig. 3 demonstrates the changes in maximum quantum yield for primary photochemistry (*ϕ*_Po_), the quantum yield for electron transport (*ϕ*_Eo_), the probability that a trapped exciton moves an electron into the electron transport chain beyond Q_A_^−^ (*ψ*_Eo_), the quantum yield for dissipated energy (*ϕ*_DIo_) in grape leaves during high temperature stress and recovery. Heat stress at 35°C did not significantly (*P*>0.05) alter *ϕ*_Po_, *ϕ*_Eo_, *ψ*_Eo_ and *ϕ*_DIo_ in grape leaves. *ϕ*_Po_ significantly declined while *ϕ*_DIo_ was enhanced at the end of first and second heat stress of 40°C and 45°C. However, at the same time, *ϕ*_Eo_ and *ψ*_Eo_ showed no change at 40°C, but decreased at 45°C compared with the control. *ϕ*_Po_ decreased and *ϕ*_DIo_ rose at 40°C less than at 45°C at the first stress. However, *ϕ*_Po_ and *ϕ*_DIo_ at 40°C was similar to those at 45°C at the second stress. After both stress periods, these parameters recovered to control levels by the first day (Day 2 and Day 3) of recovery.

**Figure 3:** Acceptor parameters (*ϕ*_Po_, *ϕ*_Eo_, *ψ*_o_ and *ϕ*_DIo_) of PSII in grape leaves under different heat treatments and following recovery. 25°C: normal growth and recovery temperature; 35, 40 and 45°C: high temperature treatments. Each value represents the mean ± S.E. of four replicates. At the same time point, the numerical values with different letters are significantly different (*P*<0.05) according to Duncan's multiple comparison.

*δ*_Ro_ expresses the redox state of PSI, i.e., the efficiency with which an electron from PQ through PS I to reduce PS I end electron acceptors. Heat stress at 35°C and 40°C did not change the *δ*_Ro_ in grape leaves, but the *δ*_Ro_ at 45°C rose significantly (*P*<0.05). However, these parameters recovered to control levels in the first day of recovery (Fig. 4).

**Figure 4:** Acceptor parameter *δ*_Ro_ (the efficiency with an electron can move from pq through PSI to the PSI end electron acceptor) in grape leaves under heat treatments at different levels and following recovery. 25°C: normal growth and recovery temperature; 35, 40 and 45°C: high temperature treatments. Each value represents the mean ± S.E. of four replicates. At the same time point, the numerical values with different letters are significantly different (*P*<0.05) according to Duncan's multiple comparison.

### PSII efficiency and excitation energy dissipation

PSII efficiency and excitation energy dissipation in grape leaves was examined by modulated fluorescence techniques. Fig. 5 shows that heat stress at 35°C had no effect on the actual PSII efficiency (*Φ*_PSII_), photochemical quenching coefficient (*q*_p_), as well as non-photochemical quenching (NPQ). Heat stress at 40 and 45°C led to a sharp decrease of *Φ*_PSII_ and *q*_p_, and a striking increase of NPQ. After the first 40°C stress, NPQ, *Φ*_PSII_ and *q*_p_ recovered to the control levels the following day (Day 2). With a 1 d recovery after the second 40°C stress, *Φ*_PSII_ slowly rose while NPQ declined to some extent, but *q*_p_ reached the control level. On the fourth day of recovery (Day 6), NPQ, *Φ*_PSII_ and *q*_p_ had recovered to control levels. With the 45°C stress, NPQ, *Φ*_PSII_ and *q*_p_ changed more dramatically, and recovered more slowly after the second stress although they had recovered to the control levels after the first stress.

**Figure 5:** PSII efficiency and excitation energy dissipation in grape leaves under different heat treatments and following recovery. 25°C: normal growth and recovery temperature; 35, 40 and 45°C: high temperature treatments. Each value represents the mean ± S.E. of four replicates. At the same time point, the numerical values with different letters are significantly different (*P*<0.05) according to Duncan's multiple comparison.

### The activation state of Rubisco

As shown in Fig. 6, heat stress at 35°C had no influence on the activation state of Rubisco in grape leaves compared with 25°C. When the grape leaves were exposed to 40 or 45°C the first time, the Rubisco activation state declined significantly (*P*<0.05), and 45°C led to the bigger decline. However, after 1 d of recovery, the Rubisco activation state recovered to the control level. When these grape leaves were exposed to 40 or 45°C a second time, the Rubisco activation state declined more than after the first stress, with 45°C resulting in a sharper decrease. On the first day during the second recovery (Day 3), the Rubisco activation state of both treatments had not recovered to the control level although the 40°C treatment recovered more rapidly than the 45°C treatment. On Day 6, the Rubisco activation state of both the 40°C and 45°C treatments reached the control level.

**Figure 6:** The activation state of Rubisco in grape leaves under different heat treatments and following recovery. 25°C: normal growth and recovery temperature; 35, 40 and 45°C: high temperature treatments. Each value represents the mean ± S.E. of four replicates. At the same time point, the numerical values with different letters are significantly different (*P*<0.05) according to Duncan's multiple comparison.

## Discussion

The step limiting photosynthesis at high temperatures has been debated recently. One proposed limitation is heat-induced deactivation of Rubisco [12], [13], [34], [35]. The other proposed limitation is impairment of the entire electron transport chain [36], [37], [38], [39]. In fact, different high temperatures may have different effects. This study clearly shows that *P*_n_ was not limited at 35°C in grape leaves, but it was limited at 40°C and 45°C. This result is similar to views that the optimum temperature for photosynthesis is between 25 and 35°C for some grape leaves [16], [17]. When the grape leaves were stressed at 40°C or 45°C, *P*_n_ and the activation state of Rubisco were markedly reduced while *C*_i_ increased, indicating that the inhibition of photosynthesis is non-stomatal and associated with Rubisco (Fig. 1 and 6). The reduction of *P*_n_ increase proportionally with the increasing of treatment temperature. However, when the grape leaves had recovered from heat stress, the increase of *P*_n_ was accompanied by increases of *g*_s_ and the activation state of Rubisco, indicating that *P*_n_ recovery was also associated with stomatal factors and the activation state of Rubisco (Fig. 1 and 6). Recent studies with cotton, wheat, tobacco, and maize have confirmed earlier observations that Rubisco is deactivated markedly in response to moderate heat stress [12], [13], [14], [40], [41]. However, heat stress at 35°C did not significantly (*P*>0.05) influence the activation state of Rubisco in grape leaves, which is similar to the effect on *P*_n_ (Fig. 6). It has been shown that the inhibition of Rubisco activation by moderately elevated temperatures up to 40°C was fully reversible after the heated leaves were incubated at 22.5°C for 15 min [34], [42]. In the present study, Rubisco following treatment at 40°C recovered more rapidly than when treated at 45°C.

The decrease of *P*_n_ under heat stress and increase of *P*_n_ during recovery was also associated with electron transport capacity. Figs. 2, 3, 4, and 5 show that the PSII and PSI were damaged. In addition, the relationship between *P*_n_ and electron transport chain was dependent on temperature. Sage and Kubien [43] thought that it has been difficult to pinpoint specific limiting steps that control the temperature response of electron transport chain. However, the OJIP test may be used to demonstrate the limiting steps of electron transport of photosynthesis [44]. At present, the mechanism causing the decline in the electron transport rate above the thermal optimum remains uncertain. Inactivation of the oxygen-evolving complex (OEC) is implicated as a cause of heat–induced reduction in electron transport capacity, particularly at high temperatures (above 38°C in potato and above 40°C in spinach) [3], [6]. However, at moderately warm temperatures, this lesion is probably not significant, as leaves can readily alter PSII properties to reduce heat sensitivity of the OEC [3]. The present results showed that 35°C did not result in damage to OEC. Heat stress can influence the PSII reaction center, and the density of RC_QA_ may reflect the density of Q_A_-reducing PSII reaction centers [45]. In the present study, during the heat stress at 40 or 45°C and the following recoveries, changing trends of W_K_ and RC_QA_ values almost corresponded to that of *P*_n_ (Fig. 2). This indicated that heat stress and recovery influenced *P*_n_ partially via the donor side (the oxygen-evolving complex) and reaction center of PSII. Moreover, the higher stress temperature led to a slower recovery of *P*_n_.

In these experiments, *ϕ*_Po_ declined and *ϕ*_DIo_ increased at 40°C or 45°C. However, after 1 d of recovery, they returned to control levels. Interestingly, *ψ*_Eo_ and *ϕ*_Eo_ significantly (*P*<0.05) decreased in grape leaves at 45°C but 40°C had almost no influence on *ϕ*_Eo_ and *ψ*_Eo_ (Fig. 3). *ϕ*_DIo_ demonstrates the quantum yield for dissipated energy. In this study, heat stress at 40 or 45°C increased *ϕ*_DIo_. However, *ϕ*_DIo_ recovered to control levels after some time. In addition, *δ*_Ro_ represents the efficiency with which an electron can move from PQ through PSI to the PSI end electron acceptor. The differential response of the *δ*_Ro_ suggests that the redox state of PQ-pool was affected by the heat stress at 45°C but not 40°C (Fig. 4).

The efficiency of PSII under steady-state irradiance (*Φ*_PSII_) was closely related to the *P*_n_ [46]. In this study, under heat stress at 40°C or 45°C *Φ*_PSII_ and *q*_p_ decreased while NPQ increased. This suggests more energy was partitioned to heat dissipation and less energy was used in CO_2_ fixation under heat stress at both temperatures. However, the influence at 40°C was less than that at 45°C. After the second recovery, *Φ*PSII at 40°C increased more rapidly accompanied by an increase of *q*_p_ and a decline of NPQ than that at 45°C. A NPQ increase of PSII is widely observed at temperatures where electron transport capacity slows with rising temperature [34], [36], which corresponds to the change in *ϕ*_DIo_.

### Conclusions

Heat treatment at 35°C did not significantly (*P*<0.05) influence grapevine photosynthesis. The decrease of *P*_n_ in grape leaves exposed to heat stress (40 or 45°C) was mainly attributed to the activation state of Rubisco and the donor side and the reaction center of PSII. However, the increase of *P*_n_ in grape leaves following heat stress was also associated with a stomatal responsec. The acceptor side of PSII in grape leaves was responsive but less sensitive to heat stress.

## Materials and Methods

### Plant materials and treatments

One-year old ‘Zuoyouhong’ grapevines (*Vitis amurensis* L.) were planted in pots, then grown in a greenhouse at 70–80% relative humidity, 25/18°C day/night cycle, with the maximum photosynthetically active radiation at about 1,000 µmol photons m^2^ s^−1^.

The progress of the experiment is shown in Table 1. Grapevines with identical growth (10 leaves) were acclimated for two days in a controlled environment room (70–80% relative humidity, 25/18°C day/night cycle and 800 µmol m^2^ s^−1^) and divided into four groups. On the following day (the first day of the experiment, Day 1), chlorophyll fluorescence and gas exchange parameters were analyzed at 9:30 h for all plants. Then, one group of grapevines was kept at 25°C in this controlled environment room. The other three groups were treated at 35, 40 or 45°C, respectively, in controlled environment rooms (except for temperature, the other conditions were the same as the 25°C room) until 14:30 h, when the relative photosynthesis parameters were then rapidly measured. The stressed grapevines were then allowed to recover at 25°C, with the other conditions the same as before heat treatments. On day 2, the same parameters were measured at 9:30 h, then the grapevines were stressed a second time until 14:30 h, when the relative photosynthesis parameters were then rapidly measured. The treated plants were again allowed to recover at 25°C as above. Chlorophyll florescence and gas exchange parameters were measured at 9:30 h on Day 3 and Day 6 during the following four days of recovery. All of the above measurements were made on the sixth leaf from the top of each plant. The experiment process is in Table 1. Four replications were made with leaves from different grape plants.

**Table 1:** Sequence of experimental treatments.

Sequence	Actions
Day 1 9:30 h	Measure photosynthesis parameters, start heat treatment
Day 1 9:30–14:30 h	Heat treatment
Day 1 14:30 h	Measure photosynthesis parameters, end the heat treatment, then start recovery
Day 2 9:30 h	Measure photosynthesis parameters, start heat treatment
Day 2 9:30–14:30 h	Heat treatment
Day 2 14:30 h	Measure photosynthesis parameters, end heat treatment , then start recovery
Day 3–6	Recovery
Day 3 and 6 9:30 h	Measure photosynthesis parameters

### Analysis of photosynthetic gas exchange parameters

Photosynthetic gas exchange was analyzed with a Li-Cor 6400 portable photosynthesis system (Li-Cor Inc., Lincoln, NE, USA) which can control photosynthesis by means of photon flux density (PPFD), leaf temperature and CO_2_ concentration in the cuvette. Net photosynthetic rate (*P*_n_), stomatal conductance (*g*_s_) and substomatal CO_2_ concentration (*C*_i_) were determined at a concentration of ambient CO_2_ (360 µmol mol^−1^) , a PPFD of 800 µmol photons m^−2^ s^−1^, a 6 cm^2^ leaf area, a 500 µmol s^−1^ flow speed and at the treatment temperature.

### Chlorophyll fluorescence quenching analysis

Chlorophyll fluorescence was measured with a FM-2 Pulse-modulated Fluorometer (Hansatech Instruments Ltd., King's Lynn, Norfolk, UK ). The maximal fluorescence level in the dark-adapted state (*F*_m_) were measured by a 0.8 s saturating pulse at 8000 µmol m^−2^ s^−1^ after 15 min of dark adaptation. When measuring the induction, the actinic light (610 µmol photons m^−2^ s^−1^) was provided for 20 s by the FMS-2 light source. The steady-state fluorescence (*F*_s_) was thereafter recorded and a second 0.8 s saturating light of 8000 µmol photons m^−2^ s^−1^ was provided to determine the maximum fluorescence in the light-adapted state (*F*_m_′). The actinic light was then turned off and the minimal fluorescence in the light-adapted state (*F*_o_′) was determined by illumination with 3 s of far red light. The following parameters were then calculated: (1) efficiency of excitation energy captured by open PSII reaction centers, *F*_v_′/*F*_m_′ = (*F*_m_′−*F*_o_′)/*F*_m_′; (2) the photochemical quenching coefficient, *q*_p_ = (*F*_m_′−*F*_s_)/(*F*_m_′−*F*_o_′); (3) the actual PSII efficiency, ΦPSII = (*F*_m_′−*F*_s_)/*F*_m_′; and (4) non-photochemical quenching, NPQ = *F*_m_/*F*_m_′−1 [47].

### Measurement of the polyphasic rise of chlorophyll a fluorescence (O-J-I-P)

The so-called OJIP-test was employed to analyze each chlorophyll a fluorescence transient by a Plant Efficiency Analyzer (Hansatech Instruments Ltd., King's Lynn, Norfolk, UK) which could provide information on photochemical activity of PSII and status of the plastoquinone pool [48]. The transients were induced by red light of about 3000 µmol photons m^−2^ s^−1^ provided by an array of six light emitting diodes (peak 650 nm). The fluorescence signals were recorded within a time span from 10 µs to 1 s with a data acquisition rate of 10 µs for the first 2 ms and every 1 ms thereafter. The fluorescence signal at 50 µs was considered as a true *F*_o_. The following data from the original measurements were used: maximal fluorescence intensity (*F*_m_); fluorescence intensity at 300 µs (*F*_k_) [required for calculation of the initial slope (*M*_o_) of the relative variable fluorescence (V) kinetics and *W*_k_]; and the fluorescence intensity at 2 ms (the J-step) denoted as *F*_j_, the fluorescence intensity at 30 ms (the I-step) denoted as *F*_i_. Terms and formulae are as follows: relative variable fluorescence intensity, *V*_t_ = (*F*_t_−*F*_o_)/(*F*_m_−*F*_o_); a parameter which represent the damage to oxygen evolving complex (OEC), *W*_k_ = (*F*_k_−*F*_o_)/(*F*_j_−*F*_o_); approximated initial slope of the fluorescence transient, *M*_o_ = 4(*F*_k_−*F*_o_)/(*F*_m_−*F*_o_); probability that a trapped exciton moves an electron into the electron transport chain beyond Q_A_^−^, *ψ*_Eo_ = *ET*_o_/*TR*_o_ = (*F*_m_−*F*_j_)/(*F*_m_−*F*_o_); maximum quantum yield of primary photochemistry at t = 0, *ϕ*_Po_ = *TR*o/ABS = *F*_v_/*F*_m_; quantum yield for electron transport (at t = 0), *ϕ*_Eo_ = *ET*_o_/ABS = (*F*_m_−*F*_j_)/*F*_m_; quantum yield at t = 0 for energy dissipation,*ϕ*_DIo_ = DIo/ABS = *F*_o_/*F*_m_; the density of Q_A_-reducing reaction centers, RC_QA_ = *ϕ*_Po_×(V_j_/*M*_o_)×(ABS/CS); and the efficiency with which an electron can move from PQ through PSI to the PSI end electron acceptors, δRo = (1−*V*_i_)/( 1−*V*_j_). From OJIP transients, the extracted parameters led to the calculation and derivation of a range of new parameters (Table 2).

**Table 2:** Summary of parameters, formulae and their description using data extracted from chlorophyll a fluorescence (OJIP) transient.

Fluorescence parameters	Fluorescence parameters Description
Extracted parameters	
*F*_t_	Fluorescence intensity at time t after onset of actinic illumination
*F*_50 µs_	Minimum reliable recorded fluorescence at 50 µs with the Handy PEA fluorimeter
*F*_k_ (F_300 µs_)	Fluorescence intensity at 300 µs
*F*_P_	Maximum recorded ( = maximum possible) fluorescence at P-step
Area	Total complementary area between fluorescence induction curve and F = Fm
Derived parameters (Selected OJIP parameters)	
*F*_o_≌*F*_50 µs_	Minimum fluorescence, when all PSII RCs are open
*F*_m_ = *F*_P_	Maximum fluorescence, when all PSII RCs are closed
*V*_j_ = (*F*_2 ms_−*F*_o_)/(*F*_m_−*F*_o_)	Relative variable fluorescence at the J-step (2 ms)
*V*_i_ = (*F*_30 ms_−*F*_o_)/(*F*_m_−*F*_o_)	Relative variable fluorescence at the I-step (30 ms)
W_K_ = (*F*_k_−*F*_o_/(*F*_j_−*F*_o_)	Represent the damage to oxygen evolving complex(OEC)
*M*_o_ = 4 (*F*_300 µs_−*F*_o_)/(*F*_m_−*F*_o_)	Approximated initial slope (in ms^−1^) of the fluorescence transient V = f(t)
Yields or flux ratios	
*ϕ*_Po_ = TR_o_/ABS = 1−(*F*_o_/*F*_m_) = *F*_v_/*F*_m_	Maximum quantum yield of primary photochemistry at t = 0
*ϕ*_Eo_ = ET_o_/ABS = (*F*_v_/*F*_m_)×(1−*V*_j_)	Quantum yield for electron transport at t = 0
*ψ*_Eo_ = ET_o_/TR_o_ = 1−*V*_j_	Probability (at time 0) that a trapped exciton moves an electron into the electron transport chain beyond Q_A_^−^
*ϕ*_DIo_ = DI_o_/ABS = 1−*ϕ*_Po_	Quantum yield at t = 0 for energy dissipation
*δ*_Ro_ = REo/ETo = (1−*V*_i_)/(1−*V*_j_)	Efficiency with which an electron can move from the PQ through PSI to the PSI end electron acceptors
Density of reaction centers. RC_QA_ = *ϕ*_Po_×(ABS/CS_m_)×(*V*_j_/*M*_o_)	Amount of active PSII RCs (Q_A_-reducing PSII reaction centers) per CS at t = m

### Extraction and assay of Ribulose-1,5-bisphosphate carboxylase/ oxygenase (Rubisco, EC4.1.1.39)

Leaves disks (1 cm^2^ each) were taken, then frozen in liquid nitrogen, and stored at −80°C until assay. Rubisco was extracted according to Chen and Cheng [49]. Three frozen leaves disks were ground with a pre-cooled mortar with 1.5 ml extraction buffer containing 50 mM Hepes-KOH (pH 7.5), 10 mM MgCl_2_, 2 mM EDTA, 10 mM dithiothreitol (DDT), 1% (v/v) Triton X-100, 1% (w/v) bovine serum albumin (BSA), 10% (v/v) glycerol, 0.5 mM phenylmethylsulfonyl fluoride (PMSF), and 5% (w/v) insoluble polyvinylpolypyrrolidone (PVPP). The extract was centrifuged at 13,000×g for 5 min in an Eppendorf microcentrifuge at 2°C, and the supernatant was used immediately for enzyme assays.

For Rubisco initial activity, a 50 µl sample extract was added to a semimicrocuvette containing 900 µl of an assay solution, immediately followed by adding 50 µl 0.5 mM RuBP, mixing well. The change of absorbance at 340 nm was monitored for 40 s. For Rubisco total activity , 50 µl 0.5 mM RuBP was added 15 min after a sample extract was combined with assay solution to activate all the Rubisco. Rubisco activation state was calculated as the ratio of initial activity to total activity [49], [50].

### Statistical analyses

Data were processed with SPSS 13.0 for Windows, and each value of the means and standard errors in the figures represents four replications. Differences were considered significant at a probability level of *P*<0.05 by Duncan's multiple comparison.
